# Exosomal miR-200c suppresses chemoresistance of docetaxel in tongue squamous cell carcinoma by suppressing TUBB3 and PPP2R1B

This article has been retracted.

**DOI:** 10.18632/aging.103036

**Published:** 2020-04-20

**Authors:** Jun Cui, Haiyan Wang, Xiaohe Zhang, Xiaodong Sun, Jin Zhang, Jinji Ma

**Affiliations:** 1 Department of Dental Implantology, Jinan Stomatological Hospital, Jinan 250001, Shandong Province, China; 2 Department of Ultrasound, Shandong Provincial Qianfoshan Hospital, The First Hospital Affiliated with Shandong First Medical University, Jinan 250014, Shandong Province, China; 3 Department of Oral Disease Gaoxin Branch, Jinan Stomatological Hospital, Jinan 250001, Shandong Province, China

**Keywords:** tongue squamous cell carcinoma, docetaxel, chemoresistance, miR-200c, TUBB3, PPP2R1B

## Abstract

Background: Chemoresistance is the main challenge for treating tongue squamous cell carcinoma (TSCC). MiR-200c is an important regulator of chemoresistance. Exosomes are a promising molecule-delivery system for cancer treatment. Thus, this study aimed to investigate the role of miR-200c in chemoresistance of TSCC and whether exosomes could effectively deliver miR-200c to chemo-resistant cells and regulate cellular activities.

Results: The results showed that the downregulation of miR-200c increased resistance to DTX, migration, and invasion and decreased apoptosis, which was reversed by the overexpression of miR-200c. The NTECs-derived exosomes transported miR-200c to HSC-3DR, increasing the sensitivity to DTX in vitro and in vivo. Also, epithelial-to-mesenchymal transition (EMT) and DNA damage responses were involved in DTX resistance. Furthermore, miR-200c regulated DTX resistance by targeting TUBB3 and PPP2R1B.

Conclusion: Exosome-mediated miR-200c delivery may be an effective and promising strategy to treat chemoresistance in TSCC.

Methods: Docetaxel (DTX) resistant HSC-3 cells (HSC-3DR) were transfected with miR-200c lentivirus and cocultured with exosomes derived from normal tongue epithelial cells (NTECs) that were overexpressed with miR-200c. The roles of miR-200c and exosomal miR-200c in vitro and in vivo were determined by RNA-Seq, qRT-PCR, western blots, transmission electron microscopy, and flow cytometry, fluorescence, CCK8, Transwell, and wound healing assays.

## INTRODUCTION

Tongue squamous cell carcinoma (TSCC) is one of the most prevailing oral cancer types and is characterized by a high proliferation rate, metastasis, and recurrence [1]. Consequently, TSCC results in the dysfunction of speech, deglutition, as well as mastication [2]. Regarding cancer treatments, chemotherapy is one of the most effective approaches to improve clinical outcomes, such as improved prognosis, reduced distant metastasis, and inhibited tumor growth [3]. However, significant benefits from chemotherapy in patients with TSCC are currently limited due to chemoresistance, which is usually related to the failure of chemotherapy. Therefore, it is urgent to investigate the underlying mechanism of chemoresistance.

As a microtubule-directed drug, docetaxel (DTX) is a first-line anticancer drug that is commonly applied to treat several solid tumor types, such as lung cancer [4], breast cancer [5], prostate cancer [6], and TSCC [7]. Functionally, DTX exerts an inhibitory effect on cancer cell microtubule dynamics, including promoting microtubule polymerization, arresting the transition from metaphase to anaphase, initiating the spindle assembly checkpoint, and eventually facilitating apoptosis [8, 9]. In addition to apoptosis, multiple factors have been demonstrated to be essential in the development of drug resistance, including epithelial-to-mesenchymal transition (EMT), low drug penetrance induced by elevation of ATP-binding cassette transporters, aberrant DNA damage, and repair response, and disrupted metabolism [10–12]. Although much progress has been made in elucidating the underlying mechanism of DTX resistance, chemoresistance remains the primary barrier limiting the clinical efficacy of DTX.

Exosomes are membrane-bound vesicles, 40-100 nm diameter, and secreted from various cell types into the extracellular space after fusion with plasma membranes [13]. In recent years, growing evidence demonstrated that many membrane components including lipids, proteins, and nucleic acids including mRNAs and microRNAs (miRNAs) have been uncovered in the exosomal lumen [13]. Furthermore, these exosome-transferring molecules can be taken up by neighboring or distant cells and in turn, regulates cellular activities of recipient cells [14]. Therefore, this transporting role of exosomes has been regarded as essential to intercellular communication, which has brought increasing attention to studying the delivery of functioning molecules.

MiRNAs, 22-25 nucleotides in length, are a group of noncoding RNAs [15] and play an important role in the regulation of gene expression by binding to the 3’UTR region of targeting mRNA [16]. In particular, miRNAs can silence genes through either inhibition of protein synthesis or cleavage of targeting mRNAs [17]. As such, miRNAs are essential regulators in various cellular processes, including proliferation, apoptosis, autophagy, and migration [18]. As a multifunctional regulator, miR-200c participates in diverse biological processes, such as cell cycle [19], steroidogenesis [20], vasculogenesis [21], and EMT [22]. Moreover, it has been demonstrated that miR-200c is an essential and promising regulator of chemoresistance in various cancers. MiR-200c sensitizes breast cancer cells in response to DTX through the PTEN/Akt pathway [23]. In addition, miR-200c enhances the sensitivity of non-small cell lung cancer cells to cisplatin and cetuximab [24]. In pancreatic cancer stem cells, enforced expression of miR-200c inhibits the abilities of colony formation, invasion, and chemoresistance [25]. However, there are only a few reports about the role of miR-200c in TSCC chemoresistance.

Therefore, given the critical role of miR-200c in chemotherapy resistance and the promising role of exosomes in intercellular communication, we aimed to investigate the role of miR-200c in DTX resistance in TSCC and whether exosome-mediated delivery of miR-200c could be applied as an effective strategy to regulate chemoresistance in TSCC cells.

## RESULTS

### DTX resistance altered the morphology and cellular activities in HSC-3 cells

In TSCC cell lines, DTX resistance was induced by treating cells with escalating concentrations of DTX. The HSC-3 cell line exhibited the lowest IC50 value in response to DTX treatment (Figure 1A) and was used for subsequent experiments. Then, we grafted DTX-treated HSC-3 cells into nude mice to cycle DTX treatment in vivo with three passages. The DTX resistant HSC-3 cells (HSC-3DR) obtained from the third passage xenograft mice showed an IC50 of 4 μM, which was 2-fold higher than the relative clinical dose (2 μM) as previously described [26, 27] (Figure 1B). Next, we determined whether DTX resistance altered the morphology of HSC-3 cells. The HSC-3DR cells displayed reduced intercellular adhesion and cell polarity (Figure 1C). Also, HSC-3DR cells showed decreased apoptosis and upregulated abilities of migration and invasion compared to HSC-3 cells (Figure 1D–1F). The wound healing assay showed that HSC-3DR cells had higher motility than HSC-3 cells (Figure 2A). Furthermore, we observed that DTX resistance impacted the expressions of EMT-associated proteins, that is, inhibited the level of E-cadherin while promoted the expressions of N-cadherin, vimentin, and fibronectin (Figure 2B). Moreover, HSC-3DR cells expressed lower expression of nuclear γ-H_2_AX compared to HSC-3 cells, indicating DTX caused more DNA double-strand damage in HSC-3 cells. (Figure 2C). Together, DTX resistance-induced changes in morphology and the cellular activities were associated with EMT and DNA damage in HSC-3DR cells.

**Figure 1:** **Docetaxel-resistant HSC-3 (HSC-3DR) cells exhibited increased cell viability and inhibited apoptosis.** (**A**) Cell viability in response to different concentrations of DTX in tongue squamous cell carcinoma cell lines was determined by CCK8 assays. (**B**) Cell viability of HSC-3 and HSC-3DR cells in response to different concentrations of DTX was determined by CCK8 assays. (**C**) The morphology of HSC-3 and HSC-3DR cells (scale bars = 50 μm). (**D**) Apoptosis of HSC-3 and HSC-3DR cells was determined by flow cytometry. (**E**) Invasion ability of HSC-3 and HSC-3DR cells was determined by Transwell assays (scale bars = 50 μm). (**F**) Migration ability of HSC-3 and HSC-3DR cells was determined by Transwell assays (scale bars = 50 μm). Data are presented as mean ± SD. *P < 0.05, **P < 0.01, ***P < 0.001.

**Figure 2:** **Docetaxel resistance in HSC-3 cells (HSC-3DR) was associated with EMT and elevated drug efflux.** (**A**) Migration ability of HSC-3 and HSC-3DR cells was determined by wound healing assays (scale bars = 100 μm). (**B**) The expressions of EMT-associated proteins in HSC-3DR cells were determined by western blots. (**C**) The expression of nuclear γ-H_2_AX of HSC-3 and HSC-3DR cells was determined by fluorescence assays (scale bars = 10 μm). Data are presented as mean ± SD. *P < 0.05, **P < 0.01, ***P < 0.001.

### Downregulation of miR-200c was essential for DTX resistance in HSC-3 cells

In this study, we performed RNA-Seq analysis to determine the differential miRNA expression profile between HSC-3 and HSC-3DR cells, and the results were plotted in the volcano plot (Figure 3A). Then, we used qRT-PCR assay to verify the expressions of miRNAs that were found to be decreased in RNA-Seq analysis (Figure 3B). The results demonstrated that miR-200c was one of significantly decreased miRNA in HSC-3DR cells compared with HSC-3 cells. MiR-200c has been demonstrated to be essential for chemoresistance in several cancer types [25, 28]. Thus, we focused on the role of miR-200c in DTX resistance in TSCC. Next, we examined the expression of miR-200c in five TSCC cell lines and the results revealed that the level of miR-200c was lower in all five carcinoma cell lines relative to NTECs, but the HSC-3 cell line had higher expression of miR-200c than the other cell lines (Figure 3C). Also, the expression of miR-200c was significantly lower in HSC-3DR cells compared to HSC-3 cells (Figure 3D). To further investigate the function of miR-200c in DTX resistance, we overexpressed miR-200c through the miR-200c-encoding lentiviral vector (LV-200c). After transfection with LV-200c, the level of miR-200c was markedly increased in HSC-3DR cells (Figure 3E). In a series of functional experiments, forced expression of miR-200c resulted in lower cell viability (Figure 3F), elevated apoptosis (Figure 3G), and inhibited abilities of migration and invasion (Figure 3H, 3I), as well as reduced motility (Figure 4A). Furthermore, overexpression of miR-200c reversed the effect of DTX resistance on the expressions of EMT-associated proteins (Figure 4B) which led to more DNA damage in HSC-3DR cells (Figure 4C). Moreover, we investigated the effect of miR-200c on DTX in vivo by subcutaneously injecting LV-200c-transfected HSC-3DR cells into nude mice, followed by DTX treatment. The results showed that overexpression of miR-200c reduced DTX resistance in HSC-3DR cells in response to DTX treatment in vivo and mice treated with LV-200c-transfected HSC-3DR cells and DTX displayed the slowest tumor growth (Figure 4D, 4E). Therefore, these results together demonstrated that forced expression of miR-200c could sensitize HSC-3DR cells to DTX in both in vitro and in vivo.

**Figure 3:** **Downregulation of miR-200c was involved in docetaxel resistance in HSC-3 cells (HSC-3DR).** (**A**) volcano plot of RNA-Seq analysis. Red and green points represent significantly upregulated and downregulated miRNAs, respectively, according to fold change > 2 and adjusted *p* < 0.05. (**B**) Expressions of downregulated miRNAs in RNA-Seq analysis were verified by qRT-PCR. (**C**) The expression of miR-200c in tongue squamous cell carcinoma cell lines was determined by qRT-PCR. (**D**) The expression of miR-200c in HSC-3 and HSC-3DR cells was determined by qRT-PCR. (**E**) The efficiency of miR-200c-encoding lentiviral vectors in HSC-3DR cells was determined by qRT-PCR. (**F**) Cell viability in HSC-3DR cells treated with miR-200c-encoding lentiviral vector (LV-200c) was determined by CCK8 assays. (**G**) Apoptosis of HSC-3DR cells treated with miR-200c-encoding lentiviral vectors (LV-200c) was determined by flow cytometry. (**H**) Invasion ability of HSC-3DR cells treated with miR-200c-encoding lentiviral vector (LV-200c) was determined by Transwell assays (scale bars = 50 μm). (**I**) Migration ability of HSC-3DR cells treated with miR-200c-encoding lentiviral vector (LV-200c) was determined by Transwell assays (scale bars = 50 μm). Data are presented as mean ± SD. *P < 0.05, **P < 0.01, ***P < 0.001.

**Figure 4:** **Effect of miR-200c on docetaxel resistance in in vitro and in vivo.** (**A**) Migration ability of HSC-3DR cells treated with miR-200c-encoding lentiviral vectors (LV-200c) was determined by wound healing assays (scale bars = 100 μm). (**B**) The expressions of EMT-associated proteins in HSC-3DR cells treated with miR-200c-encoding lentiviral vectors (LV-200c) were determined by western blots. (**C**) The expression of nuclear γ-H_2_AX in HSC-3DR cells treated with miR-200c-encoding lentiviral vectors (LV-200c) was determined by fluorescence assays (scale bars = 10 μm). (**D**) Tumor volume of xenograft mice treated with HSC-3DR cells treated with miR-200c-encoding lentiviral vectors (LV-200c) and DTX. (**E**) Representative images of tumors. Data are presented as mean ± SD. *P < 0.05, **P < 0.01, ***P < 0.001.

### Exosomal miR-200c derived from NTECs was effectively internalized by HSC-3DR cells

To investigate whether exosomes derived from NTECs could transfer miRNA to HSC-3DR cells and regulate cellular activities in the recipient cells, we overexpressed miR-200c in NTECs by transfecting LV-200c. Next, exosomes secreted from NTECs with overexpression of miR-200c were isolated, and the characteristics of exosomes were determined. The results from electron microscopy and nanoparticle tracking analysis revealed that the isolated exosomes exhibited spherical morphology with a size of 80-200 nm (Figure 5A). Western blots showed that exosomes positively expressed exosomal markers, CD9 and CD63, while negatively expressed GM130 (Figure 5B). After coculturing with exosomes, HSC-3DR cells displayed high exosome-uptake efficiency (Figure 5C). Consequently, LV-200c-treated HSC-3DR cells and their exosomes exhibited higher levels of miR-200c than those treated with the LV-200c negative control (NC) (Figure 5D). Also, RNase treatment did not affect the expression of miR-200c in exosomes while the combination of RNase and Triton X-100 dramatically reduced the level of miR-200c (Figure 5E), indicating that the presence of miR-200c was located within the exosome and was protected by a double-layer exosomal membrane. Furthermore, the expression of miR-200c in exosome-cocultured HSC-3DR cells could be reversed by transfection with the miR-200c inhibitor (Figure 5F). Collectively, these resulted revealed that exosomes derived from NTECs with overexpression of miR-200c can effectively deliver miR-200c to HSC-3DR cells.

**Figure 5:** **Characteristics and effects of exosomes derived from normal tongue epithelial cells (NTEC) transfected with miR-200c.** (**A**) The morphology and size distribution of exosomes were determined by electron microscopy and nanoparticle tracking analysis (left figure: scale bars = 200 μm and middle figure: scale bars = 100 μm). (**B**) The expressions of exosome markers were determined by western blots. (**C**) The internalization of exosomes was determined by fluorescence assays. Blue: nuclei labeled with DAPI. Green: miR-200c-carrying exosomes labeled with PKH67. (**D**) The expression of miR-200c was determined by qRT-PCR in NTEC transfected with miR-200c-encoding lentiviral vectors (LV-200c) and their exosomes. (**E**) The expression of miR-200c was determined by qRT-PCR in exosomes treated with RNase A or the combination of RNase A and Triton X-100. (**F**) The expression of miR-200c was determined by qRT-PCR in HSC-3DR cells treated with miR-200c-carrying exosomes or miR-200c-carrying exosomes with the miR-200c inhibitor. (**G**) Cell viability was determined by CCK8 assays in HSC-3DR cells treated with miR-200c-carrying exosomes or miR-200c-carrying exosomes with the miR-200c inhibitor. Data are presented as mean ± SD. *P < 0.05, **P < 0.01, ***P < 0.001.

### Exosomal miR-200c reduced DTX resistance of HSC-3DR cells

To determine the effect of exosomal miR-200c on DTX resistance of HSC-3DR cells, CCK-8 assays revealed that HSC-3DR cells cocultured with miR-200c-overexpressing exosomes displayed reduced DTX resistance while such effect was abolished with the miR-200c inhibitor (Figure 5G). Similarly, miR-200c-overexpressing exosomes increased apoptosis (Figure 6A) while decreased migration (Figure 6B) and invasion (Figure 6C), as well as inhibited motility (Figure 7A) in HSC-3DR cells, which were reversed by the downregulation of miR-200c through transfection with the miR-200c inhibitor. Also, miR-200c-overexpressing exosomes caused more DNA damage in HSC-3DR cells by displaying a higher level of nuclear γ-H_2_AX (Figure 7B). Furthermore, HSC-3DR cocultured with miR-200c-overexpressing exosomes expressed higher levels of E-cadherin, whereas lower levels of N-cadherin, vimentin, and fibronectin, which were also reversed by the miR-200c inhibitor (Figure 7C). In addition, intratumor delivery of miR-200c-overexpressing exosomes could reverse DTX resistance in HSC-3DR cells in vivo as seen with smaller tumor sizes (Figure 7D, 7E). Taken together, the results suggested that exosomal miR-200c derived from NTECs may decrease DTX resistance of HSC-3DR cells in both in vitro and in vivo.

**Figure 6:** **MiR-200c-carrying exosomes promoted apoptosis and inhibited migration ability in docetaxel-resistant HSC-3 (HSC-3DR) cells.** (**A**) Apoptosis was determined by flow cytometry in HSC-3DR cells treated with miR-200c-carrying exosomes or miR-200c-carrying exosomes with the miR-200c inhibitor. (**B**) Invasion ability was determined by Transwell assays in HSC-3DR cells treated with miR-200c-carrying exosomes or miR-200c-carrying exosomes with the miR-200c inhibitor (scale bars = 50 μm). (**C**) Migration ability was determined by Transwell assays in HSC-3DR cells treated with miR-200c-carrying exosomes or miR-200c-carrying exosomes with the miR-200c inhibitor (scale bars = 50 μm). Data are presented as mean ± SD. *P < 0.05, **P < 0.01, ***P < 0.001.

**Figure 7:** **MiR-200c-carrying exosomes regulated docetaxel resistance in in vitro and in vivo.** (**A**) Migration ability was determined by wound healing assays in HSC-3DR cells treated with miR-200c-carrying exosomes or miR-200c-carrying exosomes with the miR-200c inhibitor (scale bars = 100 μm). (**B**) The expression of nuclear γ-H_2_AX was determined by fluorescence assays in HSC-3DR cells treated with miR-200c-carrying exosomes or miR-200c-carrying exosomes with the miR-200c inhibitor (scale bars = 10 μm). (**C**) The expressions of EMT-associated proteins were determined by western blots in HSC-3DR cells treated with miR-200c-carrying exosomes or miR-200c-carrying exosomes with the miR-200c inhibitor. (**D**) Tumor volume of xenograft mice treated with miR-200c-carrying exosomes or miR-200c-carrying exosomes with the miR-200c inhibitor. (**E**) Representative images of tumors. Data are presented as mean ± SD. *P < 0.05, **P < 0.01, ***P < 0.001.

### MiR-200c reduced DTX resistance of HSC-3DR cells through targeting TUBB3 and PP2R1B

To investigate the mechanism underlying the effect of exosomal miR-200c on DTX resistance of HSC-3DR, we first predicted the putative targeting genes of miR-200c using online bioinformatics tools. The results showed that two candidate genes, TUBB3 and PPP2R1B, were reported to be associated with chemoresistance [29, 30] and contained the binding site of miR-200c (Figure 8A). Next, we performed the dual-luciferase assay to verify the prediction from the bioinformatics analysis. The results showed that HSC-3DR cells transfected with both miR-200c mimics and luciferase vectors containing the wild-type 3’UTR of TUBB3 or PPP2R1B displayed lower luciferase activity, relative to those treated with vectors containing the mutant 3’UTR (Figure 8B, 8C). These results indicated that both TUBB3 and PPP2R1B were direct targeting genes of miR-200c. Both mRNA and protein expression of TUBB3 and PPP2R1B were inhibited by overexpression of miR-200c (Figure 8D, 8E). To further investigate the functions of TUBB3 and PPP2R1B in miR-200c-associated DTX resistance, we combined TUBB3/PPP2R1B-pcDNA3.1 vectors with wild-type (TUBB3/PPP2R1B-200c-WT)/mutant (TUBB3/PPP2R1B-200c-MUT) miR-200c sequence at the 3’UTR. Western blots revealed that HSC-3DR cells transfected with vectors containing the wild-type miR-200c sequence expressed almost negligible TUBB3/PPP2R1B, compared with those treated with vectors with mutant miR-200c (Figure 8F and 8G). In functional studies, TUBB3/PPP2R1B-200c-WT HSC-3DR cells exhibited higher levels of apoptosis (Figure 8I) and lower levels of cell viability (Figure 8H), migration (Figure 8J), invasion (Figure 8K), and motility (Figure 9A), compared to TUBB3/PPP2R1B-200c-MUT cells. Furthermore, TUBB3/PPP2R1B-200c-WT HSC-3DR cells showed more DNA damage than MUT-treated cells (Figure 9B). Lastly, we treated HSC-3DR cells with miR-200c-overexpressing exosomes and found that both protein expressions of TUBB3 and PPP2R1B were decreased and could be reversed with the miR-200c inhibitor (Figure 9C). Therefore, these results indicated that exosomal miR-200c may sensitize DTX resistant HSC-3 cells by mediating the TUBB3 and PP2R1B signaling pathways.

**Figure 8:** **MiR-200c regulated docetaxel resistance in HSC-3 (HSC-3DR) cells via targeting TUBB3 and PPP2R1B.** (**A**) Putative binding sites of miR-200c in 3’UTR of TUBB3 and PPP2R1B. (**B**) Relative luciferase activity was determined by luciferase reporter assays in HSC-3DR cells transfected with miR-200c mimics and luciferase vectors containing wild-type or mutant 3’UTR of TUBB3. (**C**) Relative luciferase activity was determined by luciferase reporter assays in HSC-3DR cells transfected with miR-200c mimics and luciferase vectors containing wild-type or mutant 3’UTR of PPP2R1B. (**D**) The mRNA expressions of TUBB3 and PPP2R1B were determined by qRT-PCR in HSC-3DR cells transfected with miR-200c-encoding lentiviral vectors (LV-200c). (**E**) The protein expressions of TUBB3 and PPP2R1B were determined by western blots in HSC-3DR cells transfected with miR-200c-encoding lentiviral vectors (LV-200c). (**F**) The protein expression of TUBB3 was determined by western blots in HSC-3DR cells transfected with TUBB3-carrying vectors with the wild-type or mutant miR-200c sequence. (**G**) The protein expression of PPP2R1B was determined by western blots in HSC-3DR cells transfected with PPP2R1B-carrying vectors with the wild-type or mutant miR-200c sequence. (**H**) Cell viability was determined by CCK8 assays in HSC-3DR cells transfected with TUBB3 or PPP2R1B-carrying vectors with the wild-type or mutant miR-200c sequence. (**I**) Apoptosis was determined by flow cytometry in HSC-3DR cells transfected with TUBB3 or PPP2R1B-carrying vectors with the wild-type or mutant miR-200c sequence. (**J**) Invasion ability was determined by Transwell assays in HSC-3DR cells transfected with TUBB3 or PPP2R1B-carrying vectors with the wild-type or mutant miR-200c sequence (scale bars = 50 μm). (**K**) Migration ability was determined by Transwell assays in HSC-3DR cells transfected with TUBB3 or PPP2R1B-carrying vectors with the wild-type or mutant miR-200c sequence (scale bars = 50 μm). Data are presented as mean ± SD. *P < 0.05, **P < 0.01, ***P < 0.001.

**Figure 9:** **MiR-200c-carrying exosomes regulated expressions of TUBB3 and PPP2R1B.** (**A**) Migration ability was determined by wound healing assays in HSC-3DR cells transfected with TUBB3 or PPP2R1B-carrying vectors with the wild-type or mutant miR-200c sequence (scale bars = 100 μm). (**B**) The expression of nuclear γ-H_2_AX was determined by fluorescence assays in HSC-3DR cells transfected with TUBB3 or PPP2R1B-carrying vectors with the wild-type or mutant miR-200c sequence (scale bars = 10 μm). (**C**) The protein expressions of TUBB3 and PPP2R1B were determined by western blots in HSC-3DR cells treated with miR-200c-carrying exosomes or miR-200c-carrying exosomes with the miR-200c inhibitor. Data are presented as mean ± SD. *P < 0.05, **P < 0.01, ***P < 0.001.

## DISCUSSION

One of the most common types of oral cancer, TSCC, causes serious health outcomes worldwide and causes high mortality [31]. As a major challenge, chemotherapy resistance currently hinders to achieve better clinical outcomes for patients with advanced cancers, including TSCC. To date, the mechanism underlying chemoresistance of cancer cells remains to be elucidated. Therefore, it is necessary and imperative to explore the mechanism behind anticancer drug resistance and to develop more effective therapeutic strategies. In this study, we elucidated miR-200c as an essential antitumor miRNA and inhibitor of cancer progression in TSCC. We found that miR-200c was downregulated in DTX-resistant HSC-3 cells and was functionally important for the suppression of DTX resistance. Also, the overexpression of miR-200c sensitized DTX response by targeting TUBB3 and PPP2R1B, resulting in the EMT and DNA damage responses of HSC-3DR cells. Meanwhile, our results demonstrated a promising strategy to promote the chemosensitivity of DTX by using exosome-mediated intercellular communication. MiR-200c-loading NTECs could package miR-200c into exosomes, and mediated miR-200c transfer to HSC-3DR cells, consequently rendering HSC-3DR more sensitive to DTX via binding TUBB3 and PPP2R1B.

MiR-200c was first discovered in several cancer cell lines due to its aberrant expression [32]. Hundreds of studies reported that miR-200c plays an important role in various biological processes, including EMT, apoptosis, cell proliferation, cell migration, as well as therapy resistance in multiple tumor types [33, 34]. Regarding chemoresistance, miR-200c, an illustrious antitumor factor, is one of the most well-documented miRNAs in terms of the regulation of chemotherapy resistance in cancers. In the present study, downregulated miR-200c was required for increased DTX resistance in HSC-3 cells, along with enhanced cell viability, migration, and invasion, and inhibited apoptosis. The similar expression patterns of miR-200c were also reported in other cancer types. For example, loss of miR-200c contributes to elevated chemotherapeutic resistance to doxorubicin in breast cancer cells, which is related to KRAS signaling [35]. Also, the suppression of miR-200c is associated with reduced sensitivity to chemotherapeutic drugs in recurrent and metastatic colorectal cancers [36]. Beyond these, it has been reported that the upregulation of miR-200c can promote the sensitivity to chemotherapeutic drugs in some cancer types. In ovarian cancer, miR-200c sensitizes tumor cells to taxane by binding to TUBB3 [37, 38]. Also, the overexpression of miR-200c is found to enhance sensitivity to cisplatin in melanoma cells [39]. Collectively, miR-200c may play essential and context-dependent roles in chemoresistance in different cancer types.

As a transformation process from immotile epithelial cells to motile mesenchymal cells, EMT changes cell-cell interactions [40]. As an important step during embryonic morphogenesis, EMT contributes to the development and progression of tumors [41]. As a complex process, EMT is characterized by the loss of cell surface marker E-cadherin and the gain of mesenchymal markers, such as N-cadherin, vimentin, and fibronectin [42]. In this study, DTX resistant HSC-3DR cells inhibited expression of E-cadherin as well as enhanced expressions of N-cadherin, vimentin, and fibronectin, indicating that EMT may participate in the development of DTX resistance in TSCC. Moreover, ZEB1, an essential EMT-related transcription factor, can modulate miR-200c-mediated feed-forward loop to promote EMT, leading to invasion of tumor cells [43]. It has also been reported that enforced miR-200c expression functions as an inhibitory factor to modulate EMT in pancreatic cancer stem cells [22]. Furthermore, miR-200c suppresses the metastatic ability of EMT in head and neck squamous cell carcinoma (HNSCC) by targeting BMI1/ZEB1. Collectively, EMT may be an essential underlying mechanism behind chemoresistance and miR-200c may be an important regulator in chemoresistance-associated EMT.

In addition to EMT, another manifestation associated with DTX resistance is DNA damage and repair. In this study, we performed a fluorescence assay to detect nuclear γ-H_2_AX expression, an indicator of DNA double-strand breaks [44], and the results revealed that HSC-3DR cells displayed less DNA damage than non-resistant cells, which was reversed by forced expression of miR-200c. Moreover, DTX treatment-induced DNA damage and repair response has been reported in gastric cancer [45]. In non-small cell lung carcinoma (NSCLC), microarray chip technology revealed that DTX resistance leads to aberrant expressions of 6 miRNAs, in which 85 targeting genes are related to DNA damage and repair responses [46]. Also, a systemic study by microarray indicated that DTX affects gene expression and function, including DNA damage responses [47]. Combining with our findings, these results suggest that DNA damage and repair responses are a primary mechanism behind DTX resistance in cancer cells.

To further investigate the mechanism underlying miR-200c-associated chemoresistance in TSCC, we performed bioinformatics analysis and a series of functional experiments to determine the targeting genes of miR-200c. Consequently, TUBB3 and PPP2R1B were found to be two critical regulators in miR-200c-related DTX resistance. Our results revealed that miR-200c displayed an inhibitory effect on the expressions of TUBB3 and PPP2R1B, whereas rescuing their expressions could reverse the roles of miR-200c in DTX resistance and cellular activities. In the past decade, both TUBB3 and PPP2R1B have been well studied in chemoresistance in various tumor types [28]. Specifically, TUBB3 plays an important role in the insensitivity to microtubule-targeting anticancer agents [37, 38], in which TUBB3 is a main (up to 85%) targeting gene of miR-200c [48]. Also, the inhibitory effect of miR-200c on TUBB3 expression is uncovered in ovarian adenocarcinoma cell lines in the modulation of chemotherapy resistance [49]. On the other hand, PPP2R1B, an inhibitor of Akt phosphorylation, is inhibited by the upregulation of miR-200c, leading to cisplatin resistance in esophageal cancers through activation of the PI3K/Akt pathway [30]. Together, as two important regulators in DTX resistance, TUBB3 and PPP2R1B may be potential target molecules for developing novel strategies against chemotherapy resistance.

In recent years, exosomes have been demonstrated to be a promising molecule-delivery tool for cancer treatment [50]. In this study, we reported that exosomes derived from miR-200-overexpressing NTECs could deliver miR-200c to DTX resistant cells in vitro and sensitize the resistant cells to DTX treatment. In vivo, intra-tumor injection of miR-200c-overexpressing exosomes significantly suppressed tumor growth in response to DTX treatment. Relatively, exosomes show higher efficacy in the antitumor processes, such as inhibition of tumor growth compared to liposomes [51]. Also, exosome-based delivery displays lower cytotoxic influences in vitro and in vivo relative to synthetic nanoparticles [52]. So far, exosomal delivery has been applied to deal with chemoresistance in several tumor types, including breast cancer [53], gastric cancer [54], glioblastoma [55], and pancreatic ductal adenocarcinoma [56]. Collectively, exosome-mediated molecule shuttles have greater application value in clinical settings and may serve as a promising approach to treat chemotherapy resistance.

In conclusion, the results demonstrate that exosome-based delivery of miR-200c effectively enhances the chemosensitivity of TSCC cells to DTX in vitro and in vivo, thus providing a potential diagnostic marker for TSCC.

## MATERIALS AND METHODS

### Cell culture

All TSCC cell lines (CAL-27, HSC-3, SAS, SCC-15, and SCC-9) were purchased from American Type Culture Collection (Manassas, VA, USA). The TSCC cells were cultured in DMEM/F12 medium (Invitrogen Life Technologies, Carlsbad, CA, USA) containing 10% fetal bovine serum (Gibco, Grand Island, NY, USA), 100 U/ml streptomycin, and 100 U/ml penicillin. Cells were cultured at 37 °C in a humidified atmosphere with 5% CO_2_. The DTX resistant HSC-3 cells (HSC-3DR) were established as previously described [26, 27]. In this study, a certain number of cells (1×10^6^) were used to extract total RNA, protein, as well as functional experiments.

### Exosome isolation and identification

Exosomes were isolated from normal tongue epithelial cells (NTECs) (1×10^6^), as previously described [57, 58]. The morphology and size of the exosomes were determined by transmission electron microscopy (TEM; JEM-1-11 microscope, JEOL, Inc., Peabody, MA, USA) as previously described [59]. Exosomes (1 μg/ml) were quantified using the BCA protein assay (Abcam Trading (Shanghai) Company Ltd., Shanghai, China) and then cocultured with HSC-3DR cells.

### Cell transfection

MiR-200c mimics and inhibitors were obtained from GenePharma Co., Ltd (Shanghai, China). MiR-200c-encoding lentiviral plasmids were purchased from Takara Bio (Takara Bio Inc. Kusatsu, Shiga Prefecture, Japan). The pcDNA3.1 vector carrying TUBB3 and PPP2R1B were purchased from Abcam (Abcam Trading (Shanghai) Company Ltd., Shanghai, China). Transfection assays were performed using the Lipofectamine™ 3000 Reagent according to the manufacturer’s instructions (Invitrogen, Carlsbad, CA, USA).

### Quantitative real-time PCR (qRT-PCR)

Total RNAs of cells (1×10^6^) and exosomes (1 μg/ml) were isolated using the RNeasy Mini kit (Qiagen, Hilden, Germany) following the manufacturer’s instructions. The qRT-PCR was performed as previously described [60] and the primers used in this study are summarized in Table 1. Data were analyzed using the 2(−ΔΔCT) method [61]. The GAPDH, U6, and miR-16 were used as reference controls for TUBB3 and PPP2R1B, cellular miR-200c, and exosomal miR-200c, respectively.

**Table 1:** QRT-PCR primer sequences.

**GENE NAME**	**PRIMER SEQUENCE**
**MIR-200C FORWARD**	5′-AGCGGTAATACTGCCGGGTA-3′
**MIR-200C REVERSE**	5′-GTGCAGGGTCCGAGGT-3′
**U6 FORWARD**	5′-CGCTTCGGCAGCACATATACTAAAATTGGAAC-3′
**U6 REVERSE**	5′-GCTTCACGAATTTGCGTGTCATCCTTGC-3′
**GAPDH FORWARD**	5′-GAGTCAACGGATTTGGTCGT-3′
**GAPDH REVERSE**	5′-GACAAGCTTCCCGTTCTCAG-3′
**MIR-16 FORWARD**	5′- TAGCAGCACGTAAATATTGGCG-3′
**MIR-16 REVERSE**	5′- TGCGTGTCGTGGAGTC-3′
**TUBB3 FORWARD**	5′-GCCTGACAATTTCATCTTT-3′
**TUBB3 REVERSE**	5′-TCACACTCCTTCCG CACCA-3′
**PPP2R1B FORWARD**	5′-GTTGTTGGTGGCAGCTTCTC-3′
**PPP2R1B REVERSE**	5′-CAGCTGGGTGTGGAATTCTT-3′

### RNA-seq analysis

Total RNAs were extracted from HSC-3 and HSC-3DR cells (1×10^6^) based on the protocol mentioned above. Total RNAs (5 μg) of each sample were subjected to the treatment to remove ribosomal RNA by using RiboMinus Eukaryote Kit (Qiagen, Hilden, Germany) following the manufacturer’s instructions. The specific RNA-Seq libraries were constructed by using NEBNext Ultra Directional RNA Library Prep Kit (NEB, Beverly, MA, USA) following the manufacturer’s instructions. The RNA-Seq assay was performed in Illumina HiSeq 2000 system (Illumina, San Diego, CA, USA). FASTQ files with output reads were used to map to the human genome (hg19 assembly) (UCSC; Santa Cruz, CA) by using TopHat [62] with the default setting. The mapped reads were then analyzed by using Cufflinks software [63] for the quantification of RNA expression. The significant differentially expressed miRNAs were visualized through Volcano Plotting between HSC-3 and HSC-3DR cells. The differentially expressed miRNAs were defined by a fold change of ≥ 2 and adjusted *P* <0.05 was regarded as statistically significant.

### Western blots

Total protein of cells (1×10^6^) or exosomes (1 μg/ml) were isolated using the cell lysis buffer (Beyotime Institute of Biotechnology, Shanghai, China). The procedure of western blots was performed as previously described [58]. The primary antibodies against E-cadherin (1:1000), N-cadherin (1:1000), vimentin (1:500), fibronectin (1:1000), CD9 (1:1000), CD63 (1:1000), GM130 (1:1000), TUBB3 (1:1000), PPP2R1B (1:1000), and GAPDH (1:5000) were obtained from Abcam (Abcam Trading Company Ltd., Shanghai, China). The intensity of protein bands was determined via Imagej software [64].

### Luciferase reporter assay

Cells were co-transfected with luciferase vectors containing miR-200c mimics and wild/mutant type 3’UTR of TUBB3 and PPP2R1B using the Lipofectamine™ 3000 Reagent according to the manufacturer’s instructions (Invitrogen, Carlsbad, CA, USA). Luciferase activity was quantified by the Dual-Luciferase® Reporter Assay System (Promega™ Corporation, Madison, WI, USA).

### Fluorescence assay

The PKH67 and 4′,6-diamidino-2-phenylindole (DAPI) (Abcam Trading Company Ltd., Shanghai, China) were used to label exosomes and cell nuclei, respectively, according to the manufacturer’s instructions. Rhodamine Secondary Antibodies (Fisher Scientific™, Waltham, MA, USA) were used to label γ-H2AX according to the manufacturer’s instructions. The stained slides were imaged by confocal laser scanning microscopy (Leica, Solms, Germany).

### Flow cytometry assay

Annexin V APC Apoptosis Detection Kit (Biogems International, Inc., Westlake Village, CA, USA) and flow cytometry assays (FACSCalibur Flow Cytometer; Marshall Scientific, Hampton, NH, USA) were used to quantify cell apoptosis according to the manufacturer’s instructions.

### Cell viability, migration, invasion, and wound-healing assay

Cell viability was assessed using the CCK8 Assay Kit (Abcam Trading (Shanghai) Company Ltd., Shanghai, China) according to the manufacturer’s instructions and quantified on a microplate reader at OD450 nm. Cell migration and invasion abilities were determined using the Transwell migration assay (Fisher Scientific™, Waltham, MA, USA) according to the manufacturer’s instructions. Wound healing assay was performed using the Wound Healing assay kit (Cell Biolabs, Inc., San Diego, CA, USA).

### Animal experiment

Male BALB/C nude mice (six-weeks-old) were purchased from The Jackson Laboratory (Bar Harbor, ME, USA). The HSC-3DR cells (1 × 10^6^) were subcutaneously injected into the right flank. One week later, the tumor sizes were about 60 mm^3^. By the second week, exosomes (5 μg) were intratumorally injected twice per week with DTX treatment (90 mg/m^2^). The tumor size was quantified twice per week. In the eighth week, mice were sacrificed and tumor volume was measured and calculated using the formula V = (L × W^2^) × 0.5.

### Statistical analysis

Statistical analysis was performed using SPSS 19.0 software (SPSS Inc, Chicago, USA) and GraphPad Prism (GraphPad Software, Inc., San Diego, CA, USA). Data are presented as mean ± SD. Mean differences between groups were determined using the two-tailed Student’s t-test. Differences were considered to be significant at *P* < 0.05.

### Ethics statement

All animal experiments were conducted according to the Health guidelines and regulations of the Management of Laboratory Animals. The protocols were approved by the Institutional Animal Care and Use Committee of Jinan Stomatological Hospital.
